The article "Targeting Brain Metastases in Patients with Melanoma" was published in 2013. Journal: Biomed Res Int.

# Targeting Brain Metastases in Patients with Melanoma

**DOI:** 10.1155/2013/186563

**Published:** 2013-12-23

**Authors:** Dionysis Papadatos-Pastos, Aspasia Soultati, Mark Harries

**Affiliations:** Medical Oncology Department, Guy's and St Thomas' NHS Foundation Trust, UK

## Abstract

Patients with brain metastases from malignant melanoma historically have a very poor outcome. Surgery and radiotherapy can be used, but for the majority of patients the disease will progress quickly. In the recent past, patients with brain metastases derived only minimal benefit from cytotoxic chemotherapy. Novel therapies that have been shown to be superior to chemotherapy in metastatic melanoma have made their way in clinic and data regarding their use in patients with treated or untreated brain metastases are encouraging. In this paper we describe the use of vemurafenib, dabrafenib, and ipilimumab in patients with melanoma disseminated to the brain in addition to other treatments currently in development.

## 1. Introduction

The incidence of melanoma is steadily increasing worldwide, especially in young individuals, with significant socioeconomic implications [1]. Surgical excision of the primary skin lesion can be curative for those patients that have only localised disease. In patients that present with disseminated disease or who develop distant metastases post resection, treatment aims at prolonging survival and improving quality of life. The central nervous system (CNS) is a common site affected by malignant melanoma [2]. Brain metastases (BM) are treated with locoregional approaches, such as surgical resection or radiation-based therapies, where possible [3]. In selected cases with a small number of brain lesions surgical excision or stereotactic radiotherapy, as radical treatments, is possible [4]. The use of whole brain radiotherapy (WBRT) is recommended in patients with unresectable BM and satisfactory performance status or postoperatively [3]. For those for whom locoregional approaches are not recommended or have failed, systemic treatments can be considered. Until recently some evidence suggested that temozolomide (TMZ), an oral second generation alkylating agent, can be beneficial as a systemic agent in patients with BM, due to its satisfactory penetration via the blood brain barrier (BBB) to the CNS [5]. These reports were not confirmed in a randomised phase 3 clinical trial questioning the use of TMZ in patients with BM [6]. Recently, drugs targeting the constitutively active BRAF protein such as vemurafenib and immunotherapies such as ipilimumab were licensed for patients with metastatic melanoma (MM) [7, 8]. Nevertheless, data regarding their use in patients with BM are inconclusive due to the poor access of these patients to randomised clinical trials. There is still skepticism among oncologists regarding the effects of licensed systemic therapies for MM in patients with BM. In the present paper we present data that highlight the role of vemurafenib, dabrafenib, and ipilimumab in the treatment of patients with MM to the brain. We also discuss the potential use of compounds that affect the neoangiogenesis axis and explore the combination of systemic and locoregional therapies in this difficult-to-treat patient population. Finally, we discuss potential future treatment strategies including drugs currently on trials, such as trametinib and nivolumab.

The article "Targeting Brain Metastases in Patients with Melanoma" was published in 2013. Journal: Biomed Res Int.

## 2. Targeting the Mutated BRAF Protein

Approximately 40%–60% of patients diagnosed with malignant melanoma will have a mutation in the gene coding for the BRAF protein, most commonly a valine to glutamic acid substitution in the 600 position of the protein (V600E) [9]. The BRAF protein is an important part of the MAPK molecular pathway that when constantly activated in this mutated state carries growth stimuli that promote carcinogenesis [9].

Vemurafenib is a potent inhibitor of the activated BRAF (V600E) protein and is the first compound to be licensed by the American and European authorities for patients with MM bearing the V600E mutation. The approval was granted based on the results of a large randomised phase 3 trial that demonstrated the superiority of vemurafenib compared to dacarbazine as first line treatment for MM [7]. As with many registration trials, patients with CNS metastases were ineligible for the study unless they had been treated or were stable for at least three months and not requiring steroids. Assessment of response to the BM was not among the pre specified end points.

A case report of a 16-year-old girl with MM to the brain suggested that vemurafenib might have activity in the CNS [10]. To further assess the efficacy of vemurafenib in BM an open label, single arm trial was designed to evaluate the safety and efficacy of the drug in patients with metastatic melanoma with BRAF V600 mutations and nonresectable BM, pretreated with radiotherapy and/or chemotherapy [11]. All patients included in the study were young (between 24 and 48 years), had from 3 to more than 10 BM, ECOG PS 0–2, and were on dexamethasone. Preliminary results showed responses to the BM as well as to the extracranial disease in the two patients assessed. The responses to the BM were associated with an improvement in symptomatology, resulting in a reduction in both steroid and analgesic use. In conclusion, this preliminary result suggests that vemurafenib is well tolerated in symptomatic patients with melanoma metastatic to the brain and that there are early but strong indications for activity in BM.

The article "Targeting Brain Metastases in Patients with Melanoma" was published in 2013. Journal: Biomed Res Int.

Dzienis and Atkinson performed a prospective single arm study of vemurafenib in 18 patients with asymptomatic BM [12]. Nine patients had not had any prior therapy to the brain (group A), six had previous surgery and/or radiotherapy with residual disease (group B) and three patients had pretreated BM but with evidence of progression in CNS before the start of Vemurafenib and were included to group A (*n* = 9 + 3 = 12). In both cohorts response rate (RR) was 50%. Time to progression (TTP) in the brain was 21 weeks for responding and 12 weeks for nonresponding patients in group A. In group B TTP was 44 weeks and 8 weeks in responders and nonresponders, respectively.

Dabrafenib is also an inhibitor of the V600E BRAF which, as mentioned above, plays a role in the regulation of cell growth [13]. It has clinical activity with a manageable safety profile in phase 1 and 2 clinical trials, in patients with BRAF(V600)-mutated metastatic melanoma [13]. Falchook and colleagues performed a phase 1 clinical trial to assess the safety and tolerability and to establish a recommended phase 2 dose (RP2D) in patients with incurable carcinomas, especially those with MM and untreated, asymptomatic BM [13]. Half of the patients (*n* = 18) treated with the RP2D had a confirmed partial response, but more importantly nine out of 10 patients with untreated BM had a reduction of the size of their CNS lesions.

BREAK-MB is a multicentre, open-label, phase 2 trial assessing the use of dabrafenib in patients with MM and BM whose tumour has a BRAF (V600E or V600K) mutation [14]. Eligible patients had histologically confirmed BRAF-mutant melanoma and at least one asymptomatic brain metastasis. Patients were split into two cohorts: those in cohort A had not received previous local treatment for brain metastases and those in cohort B had progressive brain metastases after previous local treatments. The primary endpoint was the proportion of patients with BRAF-mutant MM who achieved a response in their intracranial lesions. 39% (*n* = 29) and 30% (*n* = 20) of the patients had a response in their CNS disease in cohorts A and B, respectively. Progression free survival (PFS) for patients with a V600E mutation was 16.1 and 16.6 weeks for cohort A and cohort B, respectively. Overall survival was similar between the two cohorts (33 weeks versus 31 weeks for cohort A and B, resp.). There were two grade 4 toxicities from the CNS: a convulsion (cohort A) and an intracranial bleed (cohort B). Overall, this study highlights the efficacy and safety of dabrafenib in patients with treated or untreated (and progressed) BM from BRAF-mutant melanoma.

The article "Targeting Brain Metastases in Patients with Melanoma" was published in 2013. Journal: Biomed Res Int.

## 3. Modulating the Immune System

The exploitation of the immune system in the treatment of melanoma is not a new concept. Until recently the trend was to consider that tumors metastasing to the CNS were not affected by immune-based therapies [15] Studies with animal models strongly debate this notion and in addition ipilimumab has been linked with immune hypophysitis and ocular autoimmunity suggesting that there is activity in the intracranial environment [16–18]. Furthermore, while antibodies are not able to pass the BBB, activated T-cells may be able to penetrate it and thus providing a rationale for the use of immune modulating treatments in patients with BM [19].

IL-2 has been assessed in many clinical trials and some centres have used it for stage 4 patients with low disease burden. A recent retrospective report suggests that IL-2 is a safe and potentially useful option in patients with BM [20]. Although there were no intracranial responses recorded the median OS for this difficult to treat patient population was 8.7 months.

Data suggest that IFN gamma is a modulator of neuronal activity, mood, sleep, and other CNS functions suggesting its intracranial activity [21]. In a recent prospective trial of pegylated interferon alpha (PIA) as treatment for stage 4 disease 47 (24%) patients experienced a clinical benefit whereas median overall survival was 9.7 months. Whether PIA has anticancer activity in the CNS is not known [22].

Ipilimumab is a fully human monoclonal antibody (IgG1) that inhibits the function of cytotoxic T cell associated antigen 4 (CTLA-4) and enhances an immune response against melanoma cells [8]. Following the results from a large randomised phase 3 trial comparing ipilimumab in combination with a glycopeptide-based vaccine or alone in pretreated patients with melanoma, it is now approved for clinical use by the American and European drug licensing authorities [8]. Patients with active or untreated BM were excluded from the trial. Weber and colleagues performed a small retrospective analysis of patients with MM and found that it is a safe and tolerable treatment for patients with asymptomatic BM [23]. To prospectively validate the use of ipilimumab in patients with BM, Margolin and colleagues designed a study including 72 patients with metastatic melanoma to the brain [24]. Patients were allocated to cohort A (*n* = 51) if they were asymptomatic and did not require steroids for symptom control or cohort B (*n* = 21) if they had symptomatic BM and were on steroids. The primary endpoint of the trial was the proportion of patients with disease control (complete response, partial response, or stable disease) after 12 weeks of treatment with ipilimumab. Nine (18%) patients and one patient (5%) in cohorts A and B, respectively, achieved disease control after completing 12 weeks on treatment. Extracranial responses were documented in 14 patients in cohort A and one patient in cohort B. The less than modest clinical benefit observed in patients receiving steroids could be because steroids partly suppress the immune response that ipilimumab produces or those patients requiring glucocorticoids to control CNS symptoms are generally thought to represent a group with more aggressive disease. It is likely that steroid dependence maybe associated with low benefit from ipilimumab. There were no unexpected toxicities but it should be noted that one patient died due to drug related colitis. Overall, ipilimumab is active in the CNS and probably more in individuals with small volume asymptomatic disease in the brain.

The article "Targeting Brain Metastases in Patients with Melanoma" was published in 2013. Journal: Biomed Res Int.

Adoptive cell therapy (ACT) is a highly complex and costly treatment that is performed in few centres worldwide. It involves isolation of tumour-specific lymphocytes from the patient, their *in-vitro* culture for many weeks, and finally their infusion back to the host that has undergone conditioning with a nonmyeloablative, lymphodepleting preparative regimen. From a total of 264 patients treated with ACT, 26 were retrospectively found to have BM, of which 17 completed the treatment protocol [25]. Seven (41%) patients had a completed response to the brain and six patients an overall response (35%). This impressive result should be interpreted with caution given the small number of highly selected patient population treated.

## 4. Targeting the Neoangiogenesis Axis

Results from the many clinical trials of bevacizumab, a humanised monoclonal IgG antibody against the circulating VEGF, used alone or in combination with chemotherapy, do not support its use in stage 4 MM. It must be noted that patients with BM were excluded from most of the bevacizumab trials due to the perceived high risk of intracranial bleed.

Similar drugs to bevacizumab, sorafenib, and sunitinib (multitargeted tyrosine kinase inhibitors with anti-angiogenesis activity) have been assessed in clinical trials with no success. Amaravadi and colleagues reported that the combination of TMZ and sorafenib significantly prolonged the progression free survival of patients with BM, but this result should be interpreted with caution as there was no comparator arm [26].

Therapies that affect the neoangiogenesis axis are not currently recommended in melanoma patients with brain metastases but data from ongoing trials are awaited with interest [27].

The article "Targeting Brain Metastases in Patients with Melanoma" was published in 2013. Journal: Biomed Res Int.

## 5. Combination Therapies

Chemotherapeutic drugs previously used for the treatment of melanoma such as dacarbazine, TMZ, and fotemustine are falling out of favour given the recent advances in immune-based and targeted therapies. Nevertheless, data suggest that the effect of immunotherapies is possibly augmented with the release of chemotherapy related antigens [28]. NIBIT-M1 is a single arm phase 2 study assessing the combination of fotemustine and ipilimumab in patients with metastatic melanoma, including in the brain [19]. 86 patients were included from which 20 had asymptomatic BM at trial entry. In total, 40 (46.5%) patients achieved disease control as did 10 (50%) patients with BM. The treatment was well tolerated and no unexpected toxicities were observed. Following this interesting result, NIBIT-M2, a randomised trial comparing ipilimumab in combination with fotemustine with fotemustine alone, has been planned.

Cytotoxic drugs have also been used in parallel with tyrosine kinase inhibitors (TKI), such as sorafenib and sunitinib. The majority of these trials with TKI, for example, the trial reported by Hauschild and colleagues, a randomised controlled phase 3 trial comparing carboplatin and paclitaxel with or without sorafenib, allow patients with stable BM to be included, but outcomes for this population are rarely presented in the final paper [29]. We encourage the prospective evaluation of the CNS disease in trials assessing novel TKIs given that the micromolecular structure can theoretically achieve better concentrations in the CSF.

Radiosurgery (RS) is now an established treatment for patients with oligometastatic disease to the brain [4]. Unfortunately a significant number of patients treated with RS will relapse. Knisely and colleagues performed a retrospective analysis of patients treated with RS followed by ipilimumab [30]. Patients that had ipilimumab had a significant increase in their overall survival, 21.3 months compared to 4.9 for those that had only RS. In addition Postow and colleagues described the abscopal effect in a patient that was treated with ipilimumab and radiotherapy [31]. The abscopal effect is a phenomenon in which local radiotherapy is associated with the regression of metastatic cancer at a distance from the irradiated site. Nevertheless, the biological mechanisms underlying this effect should be further dissected and such strategies are evaluated in prospective controlled clinical trials.

The efficacy of vemurafenib with the concomitant or prior use of stereotactic or whole-brain radiotherapy was assessed in a retrospective analysis that included 12 patients with metastatic melanoma to the brain [32]. Seven (64%) patients had a neurological improvement following treatment, whereas radiographic responses were noted in 36 (75%) of 48 index lesions with 23 (48%) complete responses and 13 (27%) partial responses. Six-month local control, freedom from new brain metastases, and overall survival were 75, 57, and 92%, respectively. Of note, one patient experienced radiation necrosis. This result suggests that vemurafenib and radiotherapy-based techniques have high efficacy and an acceptable side effect profile. Nevertheless, they need to be validated in randomised controlled clinical trials.

The article "Targeting Brain Metastases in Patients with Melanoma" was published in 2013. Journal: Biomed Res Int.

Preliminary data of the efficacy of ipilimumab and vemurafenib, when used along radiotherapy, are encouraging but more evidence is needed prior to their use in clinic.

## 6. Discussion

Systemically delivered chemotherapies have shown little benefit in patients with metastatic melanoma to the brain. In the last three years, 450 patients have been included in 9 trials assessing the use of novel therapies in patients with metastatic melanoma to the brain (Table 1). Higher response rates compared to chemotherapy, good symptom control, and acceptable toxicities have been documented in this difficult-to-treat patient population. Still many questions remain unanswered.

Melanoma cells that penetrate the BBB and seed in the intracranial environment have possibly acquired new molecular characteristics that could be targeted with existing therapies. Recently, Colombino and colleagues demonstrated that melanoma lesions in the brain have an increased incidence of mutations in the BRAF protein compared with systemic melanoma [33]. Therefore, patients with well-controlled—BRAF wild type—systemic melanoma could possibly benefit from a brain tumour biopsy. Furthermore certain features found more often in melanoma cells in the brain compared to their extracranial counterparts, such as STAT3 (regulates a number of prosurvival genes) or heparanase (increases tumor invasiveness) could be exploited by the drug development community [34–36].

The lack of information regarding the activity of newer therapies in the brain is a result of the limited access of these patients to clinical trials and the insufficient reporting of the effects of treatment to the intracranial lesions. The trend is now changing and patients with metastatic disease to the CNS are more often eligible to participate in studies, including early clinical trials. In addition, in patients with melanoma who have a high rate of intracranial spread, the prospective evaluation of BM should be integrated in trial protocol where appropriate.

Ipilimumab and vemurafenib have changed the landscape of treatment options for patients with metastatic melanoma. Although enriched, our drug armamentarium is by no means complete. Trametinib, an inhibitor of MEK—a downstream protein—of the MAPK pathway, has shown promising results in patients with MM. Flaherty and colleagues performed a phase 1/2 study of the combination of trametinib with dabrafenib [37]. After the recommended phase 2 dose was reached, a comparison with single agent dabrafenib showed impressive increase in the response rates and the progression free survival in favour of the combination arm. Whether these results would be applicable for intracranial tumours is to be seen. Nivolumab is a novel immune-based therapy that is currently under development for solid tumours including melanoma [38]. In an early phase trial the combination of Nivolumab and ipilimumab produced rapid and durable responses [38]. Again data regarding outcomes for BM are not available but expected with interest.

The article "Targeting Brain Metastases in Patients with Melanoma" was published in 2013. Journal: Biomed Res Int.

In conclusion patients with melanoma and BM are no longer devoid of systemic treatment options. Effective penetration of the BBB by pharmacological compounds remains an area of ongoing research nevertheless; superior outcomes with contemporary systemic treatments are possibly a combination of higher response rates in the brain tumours and better extracranial disease control. Newer treatments show promise and further studies are needed to establish their use in this, previously thought to be doomed, patient population.

## Figures and Tables

**Table 1:** Cinical trials of targeted or immune modulatory drugs in patients with melanoma metastatic to the brain with report PFS or OS.

Trial	Type	Number of patients (*n*)	Treatment	RR in brain *n* (%)	PFS (months)	OS (months)	Intracranial bleeding (Y/N)
Falchook et al. [13]	1-2	10	Dabrafenib	9/10 (90%)	4.2	NR	NR

Long et al. [14]	2	172 (i) 89 untreated (ii) 83 pretreated	Dabrafenib	Untreated Val600Glu: 29/74 (39.2%) Val600Lys: 1/15 (6.7%) Pretreated Val600Glu: 20/65 (30.8%) Val600Lys: 4/18 (22.2%)	Untreated Val600Glu: 16.1 Val600Lys: 8.1 Pretreated Val600Glu: 16.6 Val600Lys: 15.9	Untreated Val600Glu: 33.1 Val600Lys: 16.3 Pretreated Val600Glu: 31.4 Val600Lys: 21.9	1/172

Chu et al. [20]	Retro- spective review	8	High dose IL-2	1/8 (12.5%)	NR	6.7	NR

Margolin et al. [24]	2	72 (i) 51 asymptomatic (ii) 21 symptomatic	Ipilimumab	Asymptomatic: 8/51 (16) Symptomatic: 1/21 (5%)	Asymptomatic: 1.5 Symptomatic: 1.2	Asymptomatic: 7 Symptomatic: 3.7	0
Hong et al. [25]	Retro- spective review	26	Adoptive cell therapy	ACT-TIL: 7/17 (41%) TCR-transduced lymphocytes: 2/9 (22%)	NR	ACT-TIL: 8.5 TCR-transduced lymphocutes: 15	1/26

Amaravadi et al. [26]	2	53	Temozolomide and sorafenib	NR	3.5	8	0

Di Giacomo et al. [28]	2	20	Ipilimumab and fotemustine	11/20 (55%) disease control	4.5	13.4	NR

Knisely et al. [30]	Retro-spective review	77	Ipilimumab after radiosurgery	NR	NR	21.3	NR

Narayana et al. [32]	Retro-spective review	12	Vemurafenib	36/48 (75%)	NR	NR	4/12

Total		450					

RR: response rate, PFS: progression free survival, OS: overall survival, NR: nonreported, ACT: adoptive cell therapy, TIL: tumor-infiltrating lymphocytes, TCR: T-cell receptor.
